# Evaluation of Wear Properties of Four Bulk-Fill Composites: Attrition, Erosion, and Abrasion

**DOI:** 10.1155/2021/8649616

**Published:** 2021-11-12

**Authors:** Faeze Asadian, Zahra Shahidi, Zohreh Moradi

**Affiliations:** ^1^Department of Restorative Dentistry, Dental Faculty, Tehran University of Medical Sciences, Tehran, Iran; ^2^Department of Restorative Dentistry, Dental Faculty, Birjand University of Medical Sciences, Birjand, Iran

## Abstract

**Purpose:**

Wear and increased surface roughness are among the reasons for failure of posterior composite restorations. Considering the widespread use of bulk-fill composites in the posterior region, information about their wear resistance is imperative. The aim of this study was to compare the wear and surface roughness of four bulk-fill composite resins with a conventional composite.

**Methods:**

Thirty composite discs (4 mm × 10 mm) were fabricated from EverX Posterior (GC), X-tra fil (Voco), Filtek Bulk-Fill Posterior (3M, USA), SonicFill 2 (Kerr), and Z250 (3M) composites. The baseline weight and surface roughness of specimens were measured. For the assessment of the attrition wear, the specimens were placed in a chewing simulator (Mechatronik). pH cycling was performed to erode the composite discs. They were then placed in a tooth brushing simulator machine (Dorsa) for abrasion wear. Finally, the weight and surface roughness of the specimens were measured. Data were compared using one-way ANOVA (alpha ≤ 0.05).

**Results:**

One-way ANOVA showed that the mean weight changes were significant after attrition, abrasion, and erosion (*P* = 0.019), but changes in surface roughness were not significant (*P* ≥ 0.05). The results of Tukey's test showed no significant difference between the bulk-fill composites and Z250 regarding weight loss (*P* ≥ 0.05), but the weight loss of X-tra fil was significantly greater than that of EverX (*P* = 0.007) and Filtek Bulk-Fill (*P* = 0.005).

**Conclusions:**

Considering the limitations of this study, it appears that the wear and surface roughness of bulk-fill composites are within the acceptable range and are not different from those of a conventional composite.

## 1. Introduction

Dental composite resins have attracted the attention of patients and dentists even for posterior restorations due to favorable features such as optimal esthetics and color match, conservative tooth preparation due to the ability to bond to tooth structure, and low thermal conductivity. Lots of efforts have been made to minimize the limitations and disadvantages of composite resins [1, 2]. The advent of bulk-fill composites is one of the most important achievements in this field. Using larger-sized filler particles with lower volume percentage, decreased amount of pigments, and increased translucency and using some alternative photoinitiators increase the depth of cure in these composites and enable the application of composite in thick increments in extensive cavities. Bulk-fill composite resins can be cured in up to 4 mm thick layers with medium-intensity light irradiation for 20 s to achieve the desired mechanical properties [3].

Composite restorations are subjected to repeated mechanical forces and chemical effects in the process of mastication [4, 5]. Wear occurs as a result of application of forces higher than the mechanical strength of the composite. Occlusal wear causes loss of the anatomical shape of the composite restorations. Therefore, wear resistance of a composite resin is important for long-term success of restorations [6, 7]. For this reason, wear resistance comparable to that of natural teeth is an important requirement for dental restorative material [6, 8].

Evidence shows that two- and three-body abrasion, adhesive, and erosion wears occur at noncontact sites of restorations, while a combination of abrasion, fatigue, and adhesive wear occurs in contact areas [9, 10]. Various factors such as the filler content and filler size, resin matrix chemical composition, the quality of bond between the filler and the matrix, and proper curing of the resin matrix can affect the wear rate of composite resins [8, 9, 11]. Generally, dental composites with filler particles larger than 1 *μ*m have higher resistance to attrition wear but they have unacceptably high abrasive wear that results in the loss of the anatomical form of composite restorations [10].

Surface roughness of composite resins is determined by the inorganic filler size [12]. The larger the size of fillers lost in the process of abrasion wear, the more the surface roughness increases. Surface roughness (Ra) is one of the contributors to surface discoloration of composite restorations. Pigment adsorption is higher in rougher surfaces, resulting in color change over time [13].

In a study by Han et al. [14], Filtek Bulk-Fill flowable composite showed higher abrasive wear resistance than some conventional composite resins. Bulk-fill composites showed different wear resistance, which was generally estimated to be moderate compared with the wear resistance of conventional composites. On the other hand, Engelhardt et al. [3] reported that the abrasion resistance of flowable bulk-fill composites was not superior to that of conventional composites.

Considering the contradictory results and lack of sufficient evidence regarding the properties of novel bulk-fill composite resins and the important role of wear resistance in long-term success of restorations, this study is aimed at assessing the rate of wear and surface roughness of several bulk-fill composite resins. The null hypothesis was that the tested composite resins would have similar wear resistance and surface roughness after wear.

## 2. Materials and Methods

Table 1 presents the characteristics of the four bulk-fill composite resins and the conventional composite evaluated in this study.

Using the one-way ANOVA Power Analysis option of PASS1 software and according to the results of the study of Turssi et al. [15], effect size is equal to 0.82 and standard deviation is equal to 7 and*β* = 0.2and*α* = 0.05. Minimum sample size required for each group was calculated 6 specimens.

### 2.1. Specimen Preparation

Bulk-fill composite resins were condensed in customized plexiglass molds (4 mm depth, 10 mm diameter). A glass slide (75 × 25 × 1 mm) was placed over the mold. The composites were polymerized through the glass slide from the top for 30 s with a polywave LED curing unit (Bluephase; Ivoclar Vivadent AG, Schaan, Liechtenstein) with 385-515 nm wavelength and 1200 mW/cm^2^ light intensity, which was controlled periodically using a radiometer (Optilux 100 radiometer; Kerr SDS). To fabricate the conventional composite specimens (control group), two increments of composite, each with 2 mm thickness, were applied into the same mold and light-cured by the curing unit as explained for other specimens. Next, the upper surface of the specimens was polished with coarse, medium, and fine aluminum-oxide discs (Sof-Lex; 3M ESPE, St. Paul, MN, USA). Each disc was used for 15 s to achieve a smooth surface. A total of 30 composite discs (*n* = 6) were fabricated as such. The specimens were initially weighed each 24 h using an analytical digital scale (Hochoice, China) with an accuracy of 0.001 g, until their weight was stabilized. The baseline surface roughness was measured by a contact profilometer (TR-200; Time Group Company, USA) with 0.01 *μ*m accuracy.

### 2.2. Attrition Wear

The specimens were placed in a chewing simulator (C-S-4; SD-Mechatronik Company, Germany) (Figure 1) by means of Teflon molds such that the specimens did not move inside the molds under force application. Sound human molar teeth were also mounted in Teflon molds using acrylic resin and served as antagonists in the chewing machine (Figure 2). Next, 50 N load was applied by the device vertically on the samples and then the arm of the device made an 0.8 mm lateral movement; 250,000 force cycles, equivalent to one year of normal chewing, were applied to each specimen. In order to better simulate the oral environment, the specimens were immersed in artificial saliva while applying the force. A new natural tooth was used for wear of each composite specimen. If the tooth broke during attrition, another mounted tooth would be placed in the device.

### 2.3. Erosion Wear

Specimens then underwent pH cycling for 5 days (placed in a demineralizing solution for 6 h/day and remineralizing solution for 18 h/day). The pH of the demineralizing solution was about 4.7 and it consisted of 2 mmol Ca, 2 mmol P, and 0.075 mol acetate buffer. The pH of the remineralizing solution was about 7 and it contained 1.5 mmol Ca, 0.9 mmol P, 0.15 KCl, and 0.02 mol cacodylate buffer [16]. At the end of each day, the solutions were changed and all specimens were washed with distilled water before placing them in fresh solution.

### 2.4. Abrasion Wear

After the erosion process, the abrasion test was performed with a mechanical tooth brushing machine (Dersa Brushing Device Company, Karaj, Iran). In order to simulate the abrasive wear, the specimens were mounted in silicone with hard consistency (Figure 3) and were placed in cylindrical containers that contained a solution of 25 g Colgate toothpaste (Palmolive Company, Sao Paulo, Brazil) in 100 mL of distilled water. The device had 8 spots for the placement of toothbrush and specimens. A soft toothbrush (Oral B Expert-Soft; Proctor & Gamble, Ireland) was placed in the device such that the toothbrush head was in direct contact with the specimens, and the movement of the toothbrush was adjusted so that in each reciprocating movement, all the bristles completely contacted the surface of specimens (Figure 4). A total of 100,000 cycles of tooth brushing (corresponding to 1 year of brushing by a normal person) [17] with 1 N force were performed. The toothbrush had a horizontal back-and-forth movement. Next, the samples were washed with air-water spray for 1 min and were then placed in an ultrasonic bath for 10 min. The specimens were dried in an incubator at 37°C until the weight of the samples was stabilized. The surface roughness and weight of the specimens were measured as explained for the baseline measurements. Weight loss of the specimens which was equivalent to the total amount of abrasion, attrition, and erosion wear of the composites was separately recorded for each specimen. The results were analyzed with one-way ANOVA followed by Tukey's HSD test at 0.05 level of significance.

## 3. Results

Table 2 presents the descriptive results. One-way ANOVA showed a significant difference in the mean weight change of specimens before and after attrition, abrasion, and erosion tests (*P* = 0.019). But the surface roughness changes were not significant between the composite resins (*P* ≥ 0.05, Table 3).

Also, Tukey's HSD post hoc test (Table 4) showed insignificant difference between Z250 conventional composite and other composites in terms of weight loss. X-tra fil composite experienced significant weight loss compared with EverX (*P* = 0.016) and Filtek Bulk-Fill (*P* = 0.035). EverX and Filtek Bulk-Fill composites did not have a statistically significant difference (*P* = 0.997), and SonicFill 2 did not have a significant difference with other tested composites in terms of weight loss (*P* > 0.05).

## 4. Discussion

The present study assessed the weight and surface roughness changes of several bulk-fill composites (Filtek Bulk-Fill, EverX Posterior, SonicFill 2, and X-tra fil) in comparison with a conventional composite (Filtek Z250) after abrasion, attrition, and erosion tests.

In this study, a chewing simulator was used for the attrition test, pH cycling was performed to simulate erosion, and a tooth brushing device was used for abrasion simulation. According to the American Dental Association, the acceptable wear rate of composite resins for unlimited applications such as cusp replacement in different teeth is maximally 50 *μ*m in 6 to 18 months [18]. Also, the maximum acceptable surface roughness is 500 nm [19].

The results obtained from the surface roughness test after abrasion, attrition, and erosion tests in this study showed that although the surface roughness of specimens decreased, this reduction was not significant compared with the baseline value. The rate of surface roughness in all the tested composite resins, except X-tra fil, was less than the maximum acceptable surface roughness (500 nm).

The surface roughness results after wear in the present study were inconsistent with the results of several previous studies. Han et al. [14], Al Khuraif [20], Moraes et al. [12], and O'Neill et al. [21] evaluated the surface roughness and reported that specimens showed higher surface roughness after abrasion due to the exposure of surface fillers after the resin matrix abrasion. Also, the difference in the increase in surface roughness after abrasion can be related to the difference in the size of filler particles in different composites. In nanocomposites, the filler and the matrix are worn away simultaneously. Therefore, the increase in surface roughness following wear is lower. But in microhybrid composites with a particle size of 1 *μ*m, the resin matrix is worn away first and the fillers are exposed; thus, they show higher surface roughness [12, 22]. It appears that the difference in surface roughness after abrasion is due to the fact that in these studies, the specimens were only brushed and were not subjected to erosion and attrition.

An effective factor in increasing the surface roughness following erosion and abrasion is the water sorption by the matrix, which increases the osmotic pressure at the interface of the organic matrix and the mineral fillers and causes cracks in the surface as well as hydrolytic degradation of silane and subsequent filler separation from the surface. The reason for the increase in brushing roughness after erosion is that the fillers exposed by erosion are separated from the surface under shear forces and leave small holes on the surface, which increase the surface roughness [23].

Turssi et al. [15] showed higher surface roughness of samples subjected to pH cycling than those stored in artificial saliva and deionized water. The reason was the destruction of the matrix and formation of cavities on the composite surface due to the degradation of the resin matrix and silane as a result of acid attacks.

X-tra fil composite showed higher surface roughness than the acceptable threshold in the present study. Large fillers (even larger than 20 *μ*m) that have been used to improve light penetration and curing of this composite can be the reason for this finding [24].

The results of the present study revealed that the weight loss after wear in bulk-fill composites was not significantly different from that in the conventional composite, which is consistent with the results of Engelhardt et al. [3]. They assessed the abrasion resistance of a bulk-fill flowable composite and a conventional flowable composite and showed no difference between them in terms of abrasion resistance. This finding can be due to the fact that wear resistance is a material-dependent property that varies between different composites depending on the type of matrix and filler properties, and it is not related to the bulk-fill or conventional nature of composites [3]. However, Elmamooz et al. [25] investigated the rate of weight loss and surface roughness of two types of conventional and bulk-fill composites after brushing in an in vitro study. Contrary to the results of the present study, they showed that the surface roughness of bulk-fill composite was higher than that of conventional composite after brushing, and the highest surface roughness was related to Tetric N Ceram Bulk-Fill and X-tra fil. The greatest weight loss was recorded for Tetric N Ceram Bulk-Fill, which was due to the larger size of filler particles in this bulk-fill composite compared with Grandio conventional composite. They also mentioned that greater surface roughness after brushing of the bulk-fill composite was responsible for more material loss in this process [25].

The results of the present study showed that the rate of weight loss after wear in X-tra fil composite was significantly greater than that in EverX Posterior composite and Filtek Bulk-Fill composite. One reason may be the higher surface roughness of X-tra fil following wear, which makes it easier to remove the exposed fillers in two and three-body wears and is followed by a greater weight loss in this composite [12, 15, 26].

Shimokawa et al. [26] also reported that Admira Fusion x-tra composite experienced the highest surface roughness and weight loss after brushing and Filtek Supreme Ultra and Filtek Bulk-Fill experienced the least weight loss. They concluded that there was no correlation between the filler content and wear rate because the filler content of Admira Fusion x-tra was higher than that of Filtek Bulk-Fill. Higher wear rate of Admira Fusion x-tra was attributed to its higher rate of surface roughness after wear, which causes greater loss of material mass from the rough surface during wear. Factors such as the silanization quality of the matrix and the irregular size and shape of filler particles contribute to higher wear of this composite. However, Wang et al. [17] found no correlation between weight loss after abrasion and surface roughness.

High filler percentage of X-tra fil composite can be associated with higher wear. Hu et al. [27] showed that samples with a filler percentage of less than 60% had lower rate of two-body wear, and the wear rate rapidly increased in composites with 80-87.5% filler content. Increasing the coefficient of friction between the filler and matrix particles and the weak bond between the filler and the matrix can cause mass loss from the surface of samples with high filler content, which leads to higher surface roughness in them. However, Han et al., [14], Moraes et al. [12], Wang et al. [17], and Engelhardt et al. [3] did not report a clear relationship between higher filler content and higher wear rate.

The presence of TEGDMA monomer in X-tra fil can play a role in its wear rate and surface roughness. This monomer decreases the viscosity of the resin matrix and has higher water sorption and susceptibility to hydrolysis compared with bis-GMA and bis-EMA monomers and increases the wear and surface roughness of materials. TEGDMA is also present in the composition of Z250 composite, but the different percentage of this monomer in the two composites can be the reason for the difference in the results [20].

Filler shape is another factor that affects the wear rate. It has been shown that composites with round submicron fillers have high abrasion resistance [28]. Filler size, volume, distribution and chemical properties, resin matrix properties, and photoinitiator are among other influential factors on the wear rate [8, 14]. The glass transition temperature, at which the material changes from rigid to rubber state, affects the degree of curing of composite and subsequently its wear rate as well. There is also a correlation between the Vickers hardness number and wear rate [3].

In this study, EverX Posterior and Filtek Bulk-Fill composites showed the least amount of wear. The weight loss in these two composites was significantly different from that in X-tra fil. Low wear of EverX Posterior can be attributed to better stress transfer to the resin matrix and better stress distribution due to the presence of fibers [29]. On the other hand, Kumar et al. [30] investigated the wear resistance of several types of bulk-fill composites compared with gold. Tetric N Ceram and EverX Posterior bulk-fill composites showed higher wear than cast gold. Higher wear of EverX Posterior composite can be attributed to the length of fibers (1-2 mm) used in this composite, which is longer than the maximum length for fibers (0.6-0.8 *μ*m) and can cause wear. Hamouda et al. [31] investigated the mechanical properties of nanofilled composites. The abrasion resistance of Filtek Supreme nanofilled composite was higher than that of a hybrid composite. Smaller fillers (5-20 nm) and higher filler content can be the cause of lower wear of nanofilled composites.

The best bulk-fill composites in terms of wear resistance in this study were EverX Posterior and Filtek Bulk-Fill. X-tra fil composite showed the lowest abrasion resistance. Surface roughness decreased after wear in bulk-fill composites. The surface roughness of Z250, EverX Posterior, Filtek Bulk-Fill, and SonicFill 2 composites after wear was lower than the maximum acceptable surface roughness, while the surface roughness of X-tra fil after wear was more than the maximum acceptable surface roughness. Due to the novelty of past-like bulk-fill composites and the limited number of studies that evaluated the mechanical properties of these composites as well as the inconsistencies in the results of such studies, further investigations are required to evaluate other properties such as the fracture toughness of different types of bulk-fill composites. Also, the clinical performance and long-term survival of such restorations should be evaluated in comparison with the conventional types.

## 5. Conclusions

Considering the limitations of this study, it appears that the wear and surface roughness of bulk-fill composites are within the acceptable range and are not different from those of conventional composites; thus, bulk-fill composites can be used in posterior areas.

In this study, EverX Posterior and Filtek Bulk-Fill showed the highest wear resistance, while X-tra fil showed the lowest wear resistance. Also, surface roughness of the bulk-fill composites was not different from that of the conventional composite.

## Figures and Tables

**Figure 1:** Chewing simulator containing artificial saliva.

**Figure 2:** The prepared sample and the tooth are placed opposite each other in the chewing simulator.

**Figure 3:** Sample prepared for placement in the brushing simulator.

**Figure 4:** Samples in the brushing simulator.

**Table 1:** Properties of the tested composite resins.

Commercial brand	Composite type	Manufacturing company	Constituents	Filler percentage	Color
EverX Posterior	Short-fiber composite	GC Corp, Tokyo, Japan	Short E-glass fiber filler, barium glass, bis-GMA, PMMA, TEGDMA	74.2 wt% 53.6 vol%	Universal

Filtek Bulk-Fill Posterior	Nanofilled	3M ESPE, St. Paul, MN, USA	Nonagglomerated/nonaggregated 20 nm silica filler, nonagglomerated/nonaggregated 4 to 11 nm zirconia filler, aggregated zirconia/silica cluster filler, ytterbium trifluoride filler consisting of agglomerate 100 nm particles, ERGP-DMA, diurethane-DMA, 1,12-dodecane-DMA	76.5 wt% 58.4 vol%	A2

SonicFill 2	Nanohybrid	Kerr Co., Orange, CA, USA	Poly(oxy-1,2-ethanediyl), *α,α*′-[(1-methylethylidene)di-4, 1-phenylene]bis[*ω*-[(2-methyl-1-oxo-2-propen-1-yl)oxy]-Not available. 2,2′-ethylenedioxydiethyl dimethacrylate	81.3 wt% unreported	

X-tra fil	Hybrid	VOCO Cuxhaven, Germany	Barium-boron-alumino-silicate glass, bis-GMA, UDMA, TEGDMA	86 wt% 70.1 vol%	Universal

Filtek Z250 Universal	Microhybrid	3M ESPE, St. Paul, MN, USA	Zirconia/silica without silane treatment, bis-GMA, UDMA, bis-EMA	82 wt% 60 vol%	A2

Bis-GMA: bisphenol A-glycidyl methacrylate; PMMA: poly (methyl methacrylate); TEGDMA: triethylene glycol dimethacrylate; DMA: dimethacrylate; UDMA: urethane dimethacrylate.

**Table 2:** Weight and surface roughness changes after abrasion, attrition, and erosion tests (*n* = 6).

Composite		Minimum	Maximum	Mean	Std. deviation
Z250	Weight diff. total	-9.00	-1.00	-5.1667	3.060
	Ra. diff. total	-1.53	0.46	-0.7647	0.753
	Rq. diff. total	-1.80	0.54	-0.9149	0.888
	Rz. diff. total	-4.75	2.12	-1/6712	2.482

X-tra fil	Weight diff. total	-8.00	-7.00	-7.6667	0.516
	Ra. diff. total	-0.82	0.36	-0.3785	0.419
	Rq. diff. total	-0.99	0.50	-0.4448	0.520
	Rz. diff. total	-2.66	2.91	-0.4898	2.197

EverX	Weight diff. total	-5.00	-2.00	-3.8333	1.169
	Ra. diff. total	-0.91	0.30	-0.5132	0.425
	Rq. diff. total	-1.10	-0.03	-0.6307	0.409
	Rz. diff. total	-3.04	0.53	-1.3497	1.461

Filtek Bulk-Fill	Weight diff. total	-6.20	-2.10	-4.2167	1.468
	Ra. diff. total	-0.76	-0.09	-0.4748	0.257
	Rq. diff. total	-0.87	-0.11	-0.5535	0.347
	Rz. diff. total	-2.33	1.43	-1.2167	1.381

SonicFill2	Weight diff. total	-10.00	-4.00	-5.5000	2.345
	Ra. diff. total	-1.81	0.19	-0.7075	0.741
	Rq. diff. total	-2.25	0.23	-0.8517	0.922
	Rz. diff. total	-6.87	0.16	-2.1157	2.499

**Table 3:** Results of one-way ANOVA comparing the weight and surface roughness changes of specimens after the three wear tests (abrasion, attrition, and erosion).

ANOVA						
		Sum of squares	Df	Mean square	*F*	Sig.
Weight diff. total	Between groups	53.885	4	13.471	3.610	0.019
	Within groups	93.288	25	3.732		
	Total	147.174	29			

Ra. diff. total	Between groups	0.634	4	0.159	0.514	0.726
	Within groups	7.707	25	0.308		
	Total	8.341	29			

Rq. diff. total	Between groups	0.950	4	0.238	0.540	0.708
	Within groups	11.001	25	0.440		
	Total	11.951	29			

Rz. diff. total	Between groups	8.672	4	2.168	0.509	0.729
	Within groups	106.428	25	4.257		
	Total	115.100	29			

**Table 4:** Results of Tukey's HSD post hoc test comparing the weight loss of composite resins pairwise after abrasion, attrition, and erosion tests.

W	Z250	X-tra fil	EverX	Filtek Bulk-Fill	SonicFill 2
Z250	∗	0.198	0.754	0.911	0.998
X-tra fil	0.198	∗	0.016	0.035	0.322
EverX	0.754	0.016	∗	0.997	0.575
Filtek Bulk-Fill	0.911	0.035	0.997	∗	0.778
SonicFill 2	0.998	0.322	0.575	0.778	∗

## Data Availability

If anyone requests composite wear data of this study, corresponding author will send that with pleasure.
